# lncRNA NBR2 attenuates angiotensin II-induced myocardial hypertrophy through repressing ER stress via activating LKB1/AMPK/Sirt1 pathway

**DOI:** 10.1080/21655979.2022.2062527

**Published:** 2022-06-15

**Authors:** Cansheng Zhu, Min Wang, Xianguan Yu, Xing Shui, Leile Tang, Zefeng Chen, Zhaojun Xiong

**Affiliations:** a Department of Neurology, The Third Affiliated Hospital of Sun Yat-sen University, Guangzhou, Guangdong, China; b Department of Cardiovascular Internal Medicine, The Third Affiliated Hospital of Sun Yat-sen University, Guangzhou, Guangdong, China

**Keywords:** lncRNA NBR2, myocardial hypertrophy, angiotensin II, Endoplasmic reticulum stress

## Abstract

Myocardial hypertrophy leads to heart failure (HF), and emerging researchers have illustrated that long noncoding RNAs (lncRNAs) modulate myocardial hypertrophy. Here, we explored the role and mechanism of a novel lncRNA, NBR2, in modulating angiotensin II (Ang II)-induced myocardial hypertrophy. First, we examined plasma NBR2 levels in 25 patients with HF and myocardial hypertrophy and ten healthy donors and analyzed the correlation between NBR2 profiles and patients’ clinical indicators. In addition, the overexpression experiment of NBR2 was carried out to probe the influence of NBR2 on myocardial hypertrophy. lncRNA NBR2 was down-regulated in plasma of patients with HF and myocardial hypertrophy (vs. healthy controls), and its level was negatively correlated with cardiac function (represented by left ventricular end-diastolic diameter and left ventricular ejection fraction) and degree of myocardial hypertrophy. Besides, Ang II treatment intensified the hypertrophy of human myocardial cell lines (HCM and AC16) and curbed the NBR2 expression. Overexpressing lncRNA NBR2 alleviated Angiotension II–induced myocardial hypertrophy and declined the profiles of hypertrophic markers. Moreover, up-regulating lncRNA NBR2 weakened Ang II-mediated endoplasmic reticulum (ER) stress and activated the LKB1/AMPK/Sirt1 pathway. Interfering with the LKB1/AMPK/Sirt1 axis abated the lncRNA NBR2-mediated inhibitory effect on myocardial hypertrophy and ER stress. This study confirmed that lncRNA NBR2 dampened myocardial hypertrophy and ER stress by modulating the LKB1/AMPK/Sirt1 pathway. Our study provides the first evidence that lncRNA NBR2 is positively associated with myocardial hypertrophy.

## Highlights

- AngII induces down-regulation of lncRNA NBR2 in cardiomyocytes
- Overexpression of lncRNA NBR2 significantly inhibited AngII-induced cardiac hypertrophy
- LncRNA NBR2 significantly activated the LKB1/AMPK/SIRT1 pathway
- LncRNA NBR2 attenuated ER stress induced by Ang II

## 1. Introduction

Myocardial hypertrophy is an adaptive and compensatory mechanism for maintaining cardiac output during harmful stimuli (hemodynamic diseases such as hypertension and valvular diseases). Persistent stimulation brings about chronic hypertrophy, which can normalize wall tension and eventually cause the patient to die suddenly or suffer from significant heart failure (HF) [1,2]. The pathophysiology of hypertrophy is complex and multifactorial, as it involves multiple cellular and molecular systems. In the past few decades, noncoding RNAs (ncRNAs) have attracted great attention, and their disorders are increasingly closely associated with myocardial hypertrophy and cardiovascular diseases [3]. Hence, it’s urgent to study the molecular etiology of myocardial hypertrophy to find more effective targets for the treatment of myocardial hypertrophy.

Long noncoding RNAs (lncRNAs) are more than 200 nt long, characterized by conserved sequences and low expression profiles. lncRNAs modulate multiple biological functions at the epigenetic, transcriptional and post-transcriptional levels or directly control protein activity [4]. Recently, emerging researches have confirmed that lncRNAs are largely involved in diversified human diseases, including cardiovascular diseases, such as HF [5]. For example, lncRNA TINCR relieves Angiotensin II (Ang II)-induced myocardial hypertrophy by silencing the epigenetics of CaMKII [6]. lncRNA MEG3 is up-regulated in Ang-II-treated cardiomyocytes. Knocking down MEG3 represses Ang-II-induced myocardial hypertrophy [7]. NBR2 is a newly identified lncRNA, which is an energy stress-induced lncRNA on energy stress. NBR2 interacts with AMPK to heighten the activity of AMPK, thus forming a feed-forward loop to enhance the AMPK activation in energy stress [8]. In addition, lncRNA NBR2 regulates cancer metabolism. Current data have illustrated that glucose deficiency elevates the NBR2 profile in colorectal cancer cells, and NBR2 motivates curcumin to hamper colorectal cancer cells’ proliferation by stimulating adenosine monophosphate-activated protein kinase and choking the mTOR pathway [9]. Besides, lncRNA NBR2 impedes epithelial-mesenchymal transition (EMT) in non-small cell lung cancer (NSCLC) by modulating the Notch1 pathway [10]. It is well known that metabolic dysfunction is a hallmark of myocardial hypertrophy and HF. During HF, cardiomyocyte metabolism is converted from fatty acid oxidation to glycolysis [11]. However, the role of lncRNA NBR2 in mediating metabolic checkpoints in myocardial hypertrophy has not been fully explored.

Several changes in cardiac metabolism occur in heart failure (HF), called metabolic remodeling, including changes in substrate usage and mitochondrial dysfunction, ultimately leading to ATP deficiency and impaired contractility [12]. Adenosine monophosphate-activated protein kinase (AMPK) is an energy sensor and modulator of cardiac metabolism in normal and ischemic conditions [13]. Sirtuin 1 (Sirt1) is a nicotinamide adenine dinucleotide (NAD)-dependent deacetylase widely involved in metabolic control and mitochondrial biogenesis [14]. Liver kinase B1 (LKB1) is the dominant upstream kinase of AMPK activity. Activated AMPK amplifies ATP production by regulating key steps in glucose and fatty acid metabolism and impedes cardiac protein synthesis [15]. Several studies have manifested that high doses of resveratrol (RESV) lowers oxidative stress, ameliorates vascular function, declines high BP and prevents myocardial hypertrophy by strengthening the LKB1-AMPK-eNOS signaling [16]. Aldolase A (AldoA) blocks the AMPK signal in an LKB1- and AMP-dependent manner and aggravates ISO-induced myocardial hypertrophy [11]. These studies reveal that LKB1/AMPK is linked to myocardial hypertrophy evolvement.

Here, we discovered that overexpressing NBR2 eased Angiotensin II (Ang II)-induced myocardial hypertrophy and endoplasmic reticulum stress by activating the LKB1/AMPK/Sirt1 pathway. These findings testify that lncRNA NBR2 is a potential target for therapeutic intervention in myocardial hypertrophy.

## 2. Materials and methods

### 2.1 Clinical specimens

Thirty-five subjects were divided into the left ventricular hypertrophy (LVH) group (25 donors with left ventricular hypertrophy) and the control group (10 donors without left ventricular hypertrophy) (Table 1). Inclusion criteria for the LVH group were intel-ventricular septum end-diastolic thickness (IVSD) and/or left ventricular posterior wall depth (LVPWd) ≥1.2 cm and ejection fraction (EF) >40% on echocardiography. Patients with systolic HF, tumors, infections (acute phase), brain natriuretic peptide (BNP, >400 ng/L), Parkinson’s disease, idiopathic pulmonary fibrosis, shock or liver cirrhosis, and patients who were recently treated with interferon or phenobarbital were excluded. Whole blood was collected from the patients (fasting for 8 hours) and placed into a tube containing EDTA. The Ethics Committee of The Third Affiliated Hospital of Sun Yat-sen University approved the study, and all patients signed written informed consent.

**Table 1.** Clinical characteristics of LVH patients and healthy donors

	Control(n = 10)	LVH (n = 25)	P
Age(years)	68 ± 10	70 ± 11	0.62 1
Male/female(n/n)	4/6	14/11	0.073
Smoking,n	2(20%)	15(60%)	0.144
DM, n(%)	3(30%)	12(57.6%)	0.251
Hypertension,n(%)	4(40%)	23(92%)	0.001
ACS,n(%)	2(20%)	15(60%)	0.144
Af,n(%)	0(0%)	6(24%)	0.317
Fasting glucse(mmol/L)	5.03 ± 0.64	6.17 ± 2.23	0.1 59
SBP(mmHg)	116.3 ± 25.5	160.2 ± 31.2	0.0 04
DBP(mmHg)	72.3 ± 16.1	92.5 ± 18.1	0.0 04
HDL(mmol/L)	1.22 ± 0.37	1.16 ± 0.33	0. 641
LDL(mmol/L)	2.53 ± 0.71	2.94 ± 0.98	0. 239
BNP(ng/L)	131.4 ± 80	163.4 ± 111.0	0. 414
EF(%)	80.6 ± 4. 2	54.9 ± 7	0.001
LV(cm)	4.113 ± 0.501	4.353 ± 0.538	0. 232
LVEDD(cm)	4.56 ± 0.53	4.93 ± 0.938	0.248
LVSD(cm)	0.990 ± 0.083	1.286 ± 0.096	0.001
LVPWd (cm)	0.943 ± 0.101	1.253 ± 0.073	0.001

Note: DM = diabetes mellitus, ACS =  acute coronary syndrome, Af  =  atrial fibrillation, SBP  =  systolic blood pressure, DBP  =  diastolic blood pressure, TC  =  total cholesterol, TG  =  total glyceride, HDL = high-density lipoprotein, LDL =  low-density lipoprotein, Cr =  creatinine, CK-MB   =   creatine kinase-MB, LV   =   left ventricular diameter.

### 2.2 Cell culture and treatment

Human myocardial cell lines (HCM and AC16) were bought from the American Type Culture Collection Center (ATCC). Cells were treated with the Dulbecco modified Eagle’s medium (DMEM; Thermo Fisher Science, Inc., Waltham, MA) supplemented with 10% FBS, 1% penicillin/streptomycin (100 U/mL: 100 mg/mL) and 1% glutamine (Gln) (Thermo Fisher Science, Inc.). Afterward, cells were incubated with 5% CO_2_ at 37°C. The medium was altered once every other day. Two days later, angiotensin II (Ang II) (1 mmol/L) (Merck, Billerica, MA, USA) was added to simulate cell hypertrophy and further cultured for 48 hours.

### 2.3 Cell transfection

LKB1 shRNA negative control, LKB1 shRNA, LKB1 shRNA empty vector (NC), and pcDNA-lncRNA NBR2 (lncRNA NBR2) were provided by GenePharma Co., Ltd. (Shanghai, China). HCM and AC16 cells were inoculated in 24-well cell plates at 3 × 10^5^ cells/well and incubated at 37°C with 5%CO_2_ for 24 hours before cell transfection with Lipofectamine® 3000 (Invitrogen; ThermoFisherScientific, Inc.) following the supplier’s guidelines. The transfection validity was examined by RT-qPCR. Cells were incubated at 37°C with 5% CO_2_ for 24 hours for the subsequent test.

### 2.4 Immunofluorescent staining and measurement of cell surface area

According to previous statements [17], after fixation with 4% formaldehyde, the cells on the cover glass were permeated with PBS containing 0.1% Triton X-100 for 45 min and then blocked with 3% BSA. The cells were then incubated overnight with anti-α-Actinin (Sigma-Aldrich) away from light at 4°C. Next, the coverslip was mounted onto the glass slide using DAKO mounting medium (DAKO) plus DAPI. A quantitative digital Image analysis system (Image Pro-plus Version 7.0; Media Cybernetics, Rockville, MD) with digital cameras (Olympus IX-81, Olympus, Tokyo, Japan) was adopted. The average of 50 random cell measurements selected from three independent experiments was applied to determine the cell surface area.

### 2.5 Real-time quantitative polymerase chain reaction (RT-qPCR)

The total RNA of each group was separated with the Trizol reagent and quantified. Then, it was reversely transcribed into cDNA following the TAKARA kit instructions and amplified. Primers were synthesized by Shanghai Sangon Biotech Co., Ltd., and primer sequences were exhibited in Table 2. The reaction was made with 40 cycles of pre-denaturation at 95°C for 30s, denaturation at 95°C for 5s, and annealing/extension at 60°C for 30s. Relative expression of target genes was calculated using 2^−∆∆CT^. ∆CT = target gene -β-actin, and ∆∆ = ∆CT experiment -∆CT control.

**Table 2.** Primers and small RNA sequences

The target	Forward (5 ‘-3’)	Reverse (5 ‘-3’)
lncRNA NBR2	TAGATGAACCACCTGCCTCG	AGACAGGACATGGAGAGCTG
ANP	ATCTGATGGATTTCAAGAACC	CTCTGAGACGGGTTGACTTC
BNP	ACAATCCACGATGCAGAAGCT	GGGC CTTGGTCCTTTGAGA
β-MHC	CCTC GCAATATCAAGGGAAA	TACA GGTGCATCAGCTCCAG
GAPDH	GGGA GCCAAAAGGGTCAT	GAGT CCTTCCACGATACCAA

### 2.6 Western blot (WB)

Total proteins were obtained from HCM and AC16 cells with the RIPA lysis buffer (Beyotime Biotechnology, Shanghai, China). Protein quantification was made by the Bradford method. The samples were boiled for 5 min, cooled on ice, and centrifuged for 30s. The supernatant was then taken for polyacrylamide gel electrophoresis. Afterward, the protein was transferred to polyvinylidene fluoride (membranes) under 100 V for 1 hour. Next, the membranes were blocked with 5% skim milk at room temperature (RT) for 1 hour and incubated with the primary antibodies (1:1000) of CHOP (ab194533, Abcam, MA, USA), GRP78 (ab21685), IRE1 (ab37073), p-IRE1 (ab124945), PERK (PA5-15,305, Thermo Fisher, Shanghai, China), p-PERK (PA5-40,294,), anti-LKB1 (ab199970), anti-p-LKB1 (ab63473), anti-AMPK (ab32047), anti-p-AMPK (ab92701), anti-Sirt1 (ab189494), and anti-β-actin (ab8226) overnight at 4°C. After the membranes were cleaned with TBST twice, they were incubated with HRP-labeled secondary antibodies (Abcam) for 1 hour at RT. After being rinsed three times, the membranes were exposed with the ECL chromogenic agent (Millipore, Billerica, MA, USA), and imaged with a membrane scanner.

### 2.7 Flow cytometry

Forty-eight hours after the transfection, Ang II-treated HCM and AC16 cells were harvested with trypsin, centrifuged at 1000 rpm for 4 min, washed with buffer three times, and resuspended (cell density was 3 × 10^6^ cells/mL). Then, FITC-Annexin V and PI solution were added and incubated away from light for 15 min. Cell apoptosis was checked by flow cytometry.

### 2.8 Statistical analysis

Student’s *t* test was implemented to compare the differences between the two groups. Correlation between lncRNA NBR2 expression and left ventricular end-diastolic internal diameter (LVEDD) and left ventricular ejection fraction (LVEF) in plasma of patients with myocardial hypertrophy was ascertained using Pearson correlation analysis. The Tukey-Kramer test was employed to conduct a one-way analysis of variance for multiple groups of data. All results are expressed as mean ±SEMS. The experiment was carried out in triplicate. The GraphPad Prism software (version 8.0) was utilized for plotting. *P* < 0.05 indicated statistical significance.

## 3. Results

### 3.1 lncRNA NBR2 was down-regulated in plasma of LVH patients

We assessed the mRNA level of NBR2 with RT-qPCR and discovered that NBR2 was down-regulated in the LVH group by contrast with the Con. group (Figure 1(a)). NBR2 expression in the plasma of 25 patients with LVH and its relationship with LVEDD and LVEF were monitored by Pearson analysis. As a result, NBR2 was reversely related to LVEDD and LVEF (Figure 1(b-c)).

**Figure 1.** **lncRNA was down-regulated in plasma of LVH patients** A: The relative levels of NBR2 in plasma of healthy donors (10 cases) and LVH patients (25 cases) were determined by RT-qPCR. ***P < 0.001 (vs.Normal group). B: The correlation between the levels of NBR2 and LVEF in plasma of LVH patients was analyzed by Pearson. R^2^ = 0.5275, *P* < 0.001). C: Pearson was adopted to ascertain the relationship between NBR2 and LVEDD in plasma of LVH patients. R^2^ = 0.5495, *P* < 0.001.

### 3.2 Ang II induced down-regulation of NBR2 in cardiomyocytes and aggravated cardiomyocyte hypertrophy

To ascertain whether lncRNA NBR2 contributed to myocardial hypertrophy, we treated HCM and AC16 cells with Ang II to simulate an *in-vitro* model of myocardial hypertrophy. Cell surface area is a familiar indicator of myocardial hypertrophy. Here, cell immunofluorescence staining exhibited a substantial increase in cell surface area after Ang II treatment (Figure 2(a)). At the same time, the expression of common hypertrophy markers was examined. As expected, Ang II treatment caused significant up-regulation of atrial natriuretic peptide (ANP), brain natriuretic peptide (BNP) and β-myocardin heavy chain (β-MHC) (Figure 2(b)). Finally, we checked the NBR2 profile in HCM and AC16 cells, and the results manifested that NBR2 was down-regulated compared to the Con. group (Figure 2(c)). These results signified that Ang II contributed to cardiomyocyte hypertrophy *in vitro*. In general, NBR2 was distinctly down-regulated in Ang II–induced myocardial hypertrophy, confirming its vital role in myocardial hypertrophy.

**Figure 2.** **Ang II induced the down-regulation of NBR2 in cardiomyocytes and aggravated myocardial hypertrophy** A: Immunofluorescence staining results of HCM and AC16 cells. Cell size was measured for two groups of 50 randomized cells (n = 3 for each independent experiment; nuclei was blue; α-actinin was green). B: The mRNA expression of ANP, BNP and β-MHC in HCM and AC16 cells after 48 hours of Ang II treatment was monitored by RT-qPCR C: RT-qPCR was implemented to examine the relative levels of NBR2 in HCM and AC16 cells after 48 hours of treatment with Ang II. Data were expressed as mean ±SD (n = 3). *P < 0.01, ***P < 0.001(vs.Con).

### 3.3 Overexpressing NBR2 mitigated Ang II-induced myocardial hypertrophy

To examine the function of NBR2 in myocardial hypertrophy, we transfected HCM and AC16 with NBR2 overexpression plasmids prior to Ang II stimulation. First of all, RT-qPCR results revealed a high expression of NBR2 in the cells, indicating successful transfection (Figure 3(a)). Secondly, after the induction of cardiomyocyte hypertrophy with Ang II, cellular immunofluorescence testified that transfection of NBR2 overexpression plasmids in cardiomyocytes declined the relative cell area (Figure 3(b)). What’s more, overexpressed NBR2 hindered Ang II–induced myocardial hypertrophy, as evidenced by declined ANP, BNP, and β-MHC mRNA levels (vs. the Vector group) (Figure 3(c)). These results signified that overexpressing NBR2 restrained myocardial hypertrophy in Ang II–induced HCM and AC16 cell models. Hence, we further investigated the molecular mechanism of its potential biological function.

**Figure 3.** **Overexpressing NBR2 dramatically suppressed Ang II–induced myocardial hypertrophy** A: Relative levels of NBR2 in HCM and AC16 cells transfected with NBR2 overexpression plasmid for 48 hours were testified by RT-qPCR. B: Changes in surface area of cells treated with Ang II in the presence or absence of NBR2 overexpression plasmids (n = 3 for each independent experiment; nuclear was blue; α actin was green). (Scale, 50 μM). C: ANP, BNP and β-MHC mRNA expression levels were measured with RT-qPCR in Ang II-stimulated HCM and AC16 cardiomyocytes after NBR2 overexpression plasmid transfection. Data were expressed as mean ±SD (n = 3). **P < 0.01, ***P < 0.001(vs.Con). &*P* < 0.05, &&*P* < 0.01, &&&*P* < 0.001(vs.Vector+Ang-II).

### 3.4 NBR2 notably weakened the Ang II-induced ER stress

Intensive or sustained ER stress may lead to cell apoptosis, thereby deteriorating the hypertrophied myocardium to a failing state [18]. In this study, WB was implemented to analyze the influence of ER stress molecules, and the results illustrated that overexpressing lncRNA NBR2 distinctly choked the Ang II–induced ER stress pathway and ER stress-induced apoptosis in HCM and AC16 cells (Figure 4(a-b)).

**Figure 4.** **NBR2 notably weakened Ang II–induced ER stress** WB was performed to test ER stress protein profiles in Ang II-stimulated HCM and AC16 cardiomyocytes after NBR2 overexpression plasmid transfection B: Flow cytometry manifested that NBR2 dampened Ang II–induced apoptosis. Data were expressed as mean ±SD (n = 3). **P < 0.01, ***P < 0.001(vs.Con). &*P* < 0.05, &&*P* < 0.01, &&&*P* < 0.001 (vs.Vector+Ang-II).

### 3.5 lncRNA NBR2 activated the LKB1/AMPK/Sirt1 pathway

Previous studies have demonstrated that NBR2 is lowly expressed in Ang II–induced HCM and AC16 cells. Nevertheless, the specific mechanism remains elusive. As a key sensor of cell response to energy stress, AMPK contributes to various metabolic processes. Therefore, we probed the effects of NBR2 on the mRNA and protein levels of the LKB1/AMPK/Sirt1 pathway in HCM and AC16 cells by RT-qPCR and WB. As exhibited in Figure 5(a-d), NBR2 facilitated the mRNA expression of LKB1, AMPK and Sirt1, strengthened the phosphorylation of LKB1 and AMPK, and elevated the Sirt1 expression (Figure 5(a-d)).

**Figure 5.** **NBR2 activated the LKB1/AMPK/Sirt1 pathway** A and B: Detection of mRNA and protein levels of LKB1/AMPK/SIRT1 in Ang II-stimulated HCM cardiomyocytes after NBR2 overexpression plasmid transfection was made by RT-qPCR and WB. C and D: Expression of LKB1/AMPK/SIRT1 in Ang II-stimulated AC16 cardiomyocytes after transfection with lncRNA NBR2 overexpression plasmids was monitored by RT-qPCR and WB. Data were expressed as mean ±SD (n = 3). **P < 0.01, ***P < 0.001 (vs. Con). &&*P* < 0.01, &&&*P* < 0.001(vs.Vector+Ang-II).

### 3.6 Knocking down LKB1 inactivated the AMPK/Sirt1 pathway

To verify the role of the LKB1/AMPK/Sirt1 axis in myocardial hypertrophy, we transfected shRNA in cardiomyocytes to knock down LKB1. RT-qPCR and WB results revealed that knocking down LKB1 decreased the mRNA expression of AMPK and Sirt1, hampered the AMPK phosphorylation, and hindered the Sirt1 expression in HCM and AC16 cardiomyocytes (Figure 6(a-d)). These findings uncovered that LKB1 enhanced AMPK/Sirt1 in myocardial cells.

**Figure 6.** **Knocking down LKB1 blocked the AMPK/Sirt1 pathway activation** A and B: The LKB1/AMPK/SIRT1 expression in Ang II-stimulated HCM cardiomyocytes after knockdown of LKB1 was evaluated by RT-qPCR and WB. C and D: RT-qPCR and WB were conducted to assess the LKB1/AMPK/SIRT1 level in Ang II-stimulated AC16 cardiomyocytes after transfection with NBR2 overexpression plasmids. Data were expressed as mean ±SD (n = 3). * * *P* < 0.01, * * * *P* < 0.001, (vs Sh–NC group).

### 3.7 Knocking down LKB1 weakened the inhibition of NBR2 on myocardial hypertrophy and ER stress

The relationship between lncRNAs and the LKB1/AMPK/Sirt1 has been clearly understood, but the impact of the LKB1/AMPK/Sirt1 pathway on myocardial hypertrophy remains largely unknown. Therefore, we transfected shRNA in cardiomyocytes overexpressing NBR2 to repress LKB1 expression. WB results demonstrated that inhibiting LKB1 reduced LKB1 and AMPK phosphorylation and the Sirt1 expression (Figure 7(a)). Down-regulating LKB1 aggravated Ang II–induced myocardial hypertrophy, manifested as increased mRNA levels of ANP, BNP, and β-MHC (vs. the lncRNA NBR2 + Ang II group) (Figure 7(b)). Cell immunofluorescence illustrated that attenuating LKB1 in cardiomyocytes enlarge the relative cell area of HCM and AC16 cells (vs. the lncRNA NBR2 + Ang II group) (Figure 7(c)). Additionally, WB results manifested that LKB1 inhibition activated the Ang II–induced ER stress pathway (vs. the lncRNA NBR2+ Ang II group) (Figure 7(d)). Besides, Flow cytometry uncovered that repressing LKB1 resulted in intensified Ang II–induced apoptosis in HCM and AC16 cells (Figure 7(e)). These results hinted that inhibiting the LKB1/AMPK/Sirt1 pathway aggravated Ang II-mediated myocardial hypertrophy and ER stress.

**Figure 7.** **Dampening the LKB1/AMPK/Sirt1 pathway weakened the inhibitory effect of NBR2 on myocardial hypertrophy and ER stress** lncRNA NBR2 overexpression plasmids were co-transfected with shRNA of LKB1 into Ang II-treated HCM and AC16 cardiomyocytes. A: WB was conducted to evaluate the LKB1/AMPK/SIRT1 expression in HCM and AC16 cells. B: The mRNA expression of ANP, BNP and β-MHC in HCM and AC16 cells was checked by RT-qPCR. C: Cellular immunofluorescence staining was adopted for assaying surface area changes of HCM and AC16 cells (n = 3 for each independent experiment; nuclear was blue; α-actin was green). (Scale, 50 μM). D. WB was conducted to measure ER stress protein expression in HCM and AC16 cardiomyocytes E: Flow cytometry showed that inhibiting LKB1 hindered the anti-apoptotic impact of NBR2 on HCM and AC16 cells. Data were expressed as mean ±SD (n = 3). *P < 0.05, **P < 0.01, ***P < 0.001(vs.Con). & *P* < 0.05, && *P* < 0.01, &&& *P* < 0.001 (vs.lncRNA NBR2+ Ang-II).

## 4. Discussion

In most clinical cases, persistent cardiac stress results in LVH, which is a major risk factor of HF [19,20]. As reported, noncoding RNA (ncRNA) and the LKB1/AMPK signaling are increasingly associated with myocardial hypertrophy and cardiovascular diseases [3,21]. For example, miR-195 overexpression lowers the MO25 expression and downstream AMPK signaling, exacerbating the progression of hypertrophic cardiomyopathy [22]. However, potential mechanisms targeting the biological role of lncRNAs and LKB1/AMPK/SIRT1 in myocardial hypertrophy remain obscure. Here, we found that lncRNA NBR2 was down-regulated in the plasma of LVH patients and Ang II–induced HCM and AC16 cells. Overexpressing NBR2 significantly restrained Ang II–induced myocardial hypertrophy by motivating the LKB1/AMPK/Sirt1 pathway.

The renin-angiotensin system (RAS) is essential for cardiovascular physiology. It is well known that the main effector of RAS, Ang II, binds to the angiotensin type 1 receptor (AT1R) and heightens cell growth, proliferation, migration and oxidative stress, all of which contribute to heart and vascular remodeling [23]. Multiple studies have manifested that Ang II treatment contributes to myocardial hypertrophy and increases the production of reactive oxygen species in cardiomyocytes [24,25]. Additionally, Ang II modulates the expression of several lncRNAs in myocardial hypertrophy, including SYNE1-AS1 [26], lncRNA SNHG14 [27], and lncRNA CASC15 [28]. In this article, Ang II was applied to mediate HCM and AC16 cardiomyocytes, and it was found that Ang II-treated HCM and AC16 cells had low expression of NBR2, enlarged cell surface area, and enhanced profiles of ANP, BNP, and β-MHC.

A growing number of researches have manifested that multiple lncRNAs, including lncRNA UCA1 [29], lncRNA TINCR [6], and lncRNA MIAT [30], contribute to regulating heart development and cardiovascular disease. lncRNA NBR2 is dysregulated in diversified cancers and modulates cancer evolvement [31]. However, its role in cardiovascular diseases is rarely reported. Here, NBR2 was down-regulated in Ang II–induced HCM and AC16 cells, and overexpressing NBR2 elevated mRNA levels of ANP, BNP, and β-MHC, amplified cell surface area, and enhanced the LKB1/AMPK/SIRT1 profile. There is growing evidence that prolonged and severe ER stress leads to structural or functional abnormalities in the heart, triggering abnormal cardiac cell death [32]. Meanwhile, Ang II can notably increase ER stress genes [33]. Hence, we evaluated changes in ER stress markers and discovered that overexpressing NBR2 abated Ang II-mediated ER stress. To our knowledge, our article provides the first evidence that NBR2 is positively associated with myocardial hypertrophy.

LKB1 encodes a serine/threonine kinase that acts upstream of the AMPK superfamily [34]. Moreover, several studies have exhibited that increasing the expression of LKB1 alleviates Ang II-mediated myocardial hypertrophy. For example, CSN5 maintains the AMPK activity in cardiomyocytes by enhancing LKB1, mitigating Ang II-mediated myocardial hypertrophy [35]. RXR agonists activate the LKB1/AMPK/p70S6K pathway and regulate protein synthesis to abate LVH [36]. As reported, Sirt1, a Sirtuin family member, is mainly or exclusively located in the mitochondria. Since the regeneration of mitochondrial ATP is associated with maintaining cardiac pump function, SIRT1 has been confirmed to have a protective effect on cardiac function [37,38]. Some studies have testified that activation or attenuation of MAPK modulates cardiac energy metabolism through the Sirt1 pathway, thus mitigating or aggravating myocardial hypertrophy [39,40]. In this study, Ang II treatment of HCM and AC16 cells resulted in a significant decrease in the LKB1/AMPK/SIRT1 activity. In addition, overexpressing NBR2 facilitated the LKB1/AMPK/Sirt1 profile, thereby alleviating myocardial hypertrophy and ER stress in HCM and AC16 cells. Therefore, we posit that NBR2 hampers myocardial hypertrophy by regulating the LKB1/MAPK/SIRT1 pathway.

Overall, this study revealed that NBR2 contributes to Ang II–induced myocardial hypertrophy. NBR2 may hinder myocardial hypertrophy and ER stress in Ang II–induced HCM and AC16 cells by modulating the LKB1/MAPK/Sirt1 pathway. However, whether NBR2 can be adopted as a novel therapeutic target for relieving human myocardial hypertrophy remains to be further studied.

## Data Availability

The data sets used and analyzed during the current study are available from the corresponding author on reasonable request.
